# Elucidating the monoamine oxidase B inhibitory effect of kaurene diterpenoids from *Xylopia aethiopica*: An *in silico* approach

This article has been retracted.

**DOI:** 10.1371/journal.pone.0308021

**Published:** 2024-11-27

**Authors:** Funmilayo Gladys Famuyiwa, Rajesh B. Patil, Samson Oluwaseyi Famuyiwa, Uduak Ime Olayemi, Esther Aina Olanudun, Bhoomendra A. Bhongade, Jaiprakash N. Sangshetti, Esther Oluwatosin Shalom, Suvarna N. Vakare, Mohammed Sakib Musa, Abu Tayab Moin, Mohammad Helal Uddin, Kolade Olatubosun Faloye

**Affiliations:** 1 Department of Pharmacognosy, Faculty of Pharmacy, Obafemi Awolowo University, Ile-Ife, Nigeria; 2 Department of Pharmaceutical Chemistry, Sinhgad Technical Education Society’s, Sinhgad College of Pharmacy, Pune, Maharashtra, India; 3 Department of Chemistry, Faculty of Science, Obafemi Awolowo University, Ile-Ife, Nigeria; 4 Department of Industrial Chemistry, Faculty of Science, University of Ilesa, Ilesa, Nigeria; 5 Department of Pharmaceutical Chemistry, RAK College of Pharmacy, RAK Medical & Health Sciences University, Ras Al Khaimah, United Arab Emirates; 6 Y. B. Chavan College of Pharmacy, Dr. Rafiq Zakaria Campus, Aurangabad, (MS), India; 7 Department of Applied Chemistry and Chemical Engineering, University of Chittagong, Chattogram, Bangladesh; 8 Department of Genetic Engineering and Biotechnology, Faculty of Biological Sciences, University of Chittagong, Chattogram, Bangladesh; University of Buea, CAMEROON

## Abstract

Parkinson disease is a neurogenerative disease common in adults and results in different kinds of memory dysfuntions. This study evaluated the monoamine oxidase B (MAO-B) inhibitory potential of kaurane diterpenoids previously isolated from *Xylopia aethiopica* through comprehensive computational approaches. Molecular docking study and molecular dynamics simulation were used to access the binding mode and interaction of xylopic acid and MAO-B enzyme. The ADMET properties of the phytochemical were evaluated to provide information on its druggability. The molecular docking and molecular dynamics simulation revealed xylopic acid as potential MAO-B inhibitor due to the good binding energy elicited and stability throughout the 100 ns simulation period. The ADMET properties of the ligand showed it as a promising drug candidate. The study recommend further comprehensive *in vitro* investigation towards the development of xylopic acid as potent MAO-B inhibitor.

## 1. Introduction

Parkinson’s disease (PD) has become a common neurodegenerative disorder caused by the progressive death of dopamine nerve cells in the brain [1]. The disease affects 1% of people older than 65 years and 2.6% of people above 85 years old [2]. PD is presented with episodes of motor symptoms and memory dysfunctions such as postural instability, dementia, low mood, gait disorder, resting tremor and bradykinesia [3]. These symptoms are accompanied by non-motor symptoms like autonomic dysfunction, fatigue, sleep disturbance and depression [4]. This age-related neurologic disease may also be attributed to the over-activity of monoamine oxidases (MAOs) enzymes. MAOs are enzymes containing flavin adenine dinucleotide (FAD) that metabolizes dietary and biogenic amine together with dopamine, adrenaline and serotonin (monoamine neurotransmitters) in the peripheral and central tissues [5, 6]. The quick breakdown of these molecules results in the effectivenes of synaptic neurotransmission which is extremely important in the control of brain functions. Therefore, the deficiencies in synaptic neurotransmitters can cause various neurological disorders.

MAOs exist as different isoenzymes called monoamine oxidase A (MAO-A) and monoamine oxidase B (MAO-B) with selective substrates and inhibitors [7]. MAO-B has been identified as a major isoform of MAO responsible for dopamine degradation [8]. The enzyme is mainly resident in the platelets and glial cells, with 80% of its activity experienced within the brain as it breaks down the dopamine released into the synaptic cleft [5, 7]. As age increases, the glial cell increases, which also results in increased susceptibility to neurodegenerative diseases like PD [9].

MAO-B inhibitors are bioactive chemical compounds that inhibit the action of MAO-B by blocking dopamine catabolism leading to an increase in dopamine levels at the synaptic cleft and enhancement of dopamine signaling [10]. They also facilitate reduction in the accumulation of the products of the MAO-B metabolism of dopamine, which are hydrogen peroxide and dihydroxyacetaldehyde, which are toxic metabolites [11]. Several irreversible MAO-B inhibitors, like rasagiline and selegiline are currently prescribed as effective therapeutic agents [12]. However, these irreversible synthetic MAO-B inhibitors have several drawbacks like prolonged duration of action, target disruption and immunogenicity [13]. Therefore, it is important to investigate natural products as potential reversible MAO-B inhibitors that could be used to treat PD.

Kaurene diterpenoids are a unique category of diterpenes found in medicinal plants native to Africa and Asia [14, 15]. This class of diterpene has been isolated from *Xylopia aethiopica*, *Plectranthus asirensis*, *Annona squamosa* and *Annona glabra* [16–18]. Medicinal plants like *X*. *aethiopica* are used to treat neurodegenerative disease, and kaurane-type diterpenoids are among its major chemical constituents [19]. *Xylopia aethiopica* has been pharmacologically identified as a memory and learning enhancement, antimalarial, analgesic, neuroprotective, antidiabetic, anti-allergic, antidepressant and anti-inflammatory agent [18, 20–25].

Molecular docking and molecular dynamics simulation (MDS) are faster and cheaper methods of identifying potential drug candidates, which are predicted based on their binding energy, binding mode and interactions [26–28]. ADMET studies are useful in predicting the pharmacokinetic properties of phytochemicals that can be subjected to clinical trials [29, 30]. These computational drug discovery methods has been widely adopted due to their eco-friendly, robustness, accuracy and easy of drug candidate identification [30–33]. However, extensive use of different computational drug discovery methods could enhance the accuracy and time taken for drug design [34–36]. Despite the varieties of pharmacological studies previously performed on extractives of *X*. *aethiopica*, the MAO-B inhibitory property of its kaurene diterpenoids is yet to be investigated. Herein, we investigate the MAO-B inhibitory property of kaurane diterpenoids from *X*. *aethiopica* using molecular docking, molecular dynamics simulation, ADMET and in vitro methods.

## 2. Methods

### 2.1. Protein and ligand preparation

The 3D crystallographic structure of MAO-B enzyme with PDBID: 2V5Z [37] was retrieved from the protein data bank (www.rcsb.org) and loaded on PyMol software in order to remove the water molecules, co-factors and ions. The co-crystallized ligand (safinamide) was also identified on PyMol software and the residues within 5 Å resident at the binding site of the protein were selected. Thereafter, the co-crystallized ligand was removed to obtain a clean protein. The protein was saved in PDB format for docking purpose.

The chemical structure of *X*. *aethiopica* kaurane diterpenoids was built with Spartan 14 software (see S1 Fig), while the standard drug (rasagiline) was downloaded from the PubChem database (https://pub-chem.ncbi.nlm.nih.gov/compound/3052776). The chemical structures were saved in SDF format and loaded into Open Babel for energy minimization under the MMFF94x forcefield. Then the energy-minimized ligand were saved as PDBQT file.

### 2.2. Molecular docking studies

The docking methodology was first validated by re-docking the co-crystallized ligand in the MAO-B enzyme’s binding pocket followed by the estimation of its RMSD value.

The molecular docking studies of the phytochemicals and rasagiline against the MAO-B enzyme was done by converting the clean protein’s PDB file to PDBQT using the MGL software. Thereafter, the protein was loaded into the Autodock Vina interface of PyRx 0.8 software [38] and amino acid residues resident within 5 Å was selected. Then the grid box of the protein was adjusted to center_x = 51.0741, center_y = 155.5819, center_z = 30.0842 and size_x = 22.8706, size_y = 25.6361, size_z = 25.6808. The PDBQT file of individual phytoconstituent and rasagiline were loaded and molecular docking was carried out against MAO-B enzyme at an exhaustiveness of 100. After successfully completing the docking procedure, the binding poses of the ligand was retrieved and those with the lowest RMSD value were selected for hydrogen bonding, hydrophobic and pi-interactions analysis using the Discovery Studio Visualizer software.

### 2.3. Molecular dynamics simulations

The docked complexes of the drug candidate and Rasagiline with MAO-B and MAO-B in native form without any bound ligands (referred to here onwards as apo MAO-B) were subjected to molecular dynamics simulations. The input topology of MAO-B was prepared using the CHARMM-36 force field [39, 40] and the topology of the hit molecule and rasagiline was obtained from the CGenFF server, which uses the CHARMM General Force Field [39, 41]. During input preparation, the complexes and apo MAO-B were held in a dodecahedron unit cell and solvated with water using a TIP3P water model [42]. Subsequently, the systems were neutralized by adding counter ions where the complex of hit molecule with MAO-B and apo MAO-B systems needed 2 sodium ions, and the complex of rasagiline with MAO-B needed one sodium ion. The neutralized systems were subjected to unrestrained energy minimization until the force constant reached 100 kJ/mol norm with the steepest descent energy minimization. The systems were later subjected to equilibration initially at constant volume and temperature conditions where a temperature of 300K was achieved by a modified Berendsen thermostat [43] and later at constant volume and pressure conditions where pressure of 1 bar atmospheric pressure was achieved by Berendsen barostat [44]. Each equilibrated system was subjected to 100 ns production phase MD simulation using Gromacs 2020.4 [45] program on a remote server of the Bioinformatics Resources and Applications Facility (BRAF), C-DAC, Pune. During the production phase MD simulations, the covalent bonds were restrained with the LINCS algorithm [46] and the constant temperature and pressure conditions were achieved by a modified Berendsen thermostat and Parrinello-Rahman barostat [47], respectively. The long-range interaction energies, such as Coulomb and Lennard Jones interaction energies, were calculated using the Particle Mesh Ewald (PME) [48] method with a cutoff distance of 1.2 nm. Post-production phase MD simulations, the root mean square deviations (RMSD) in backbone atoms and ligand atoms, root mean square fluctuations (RMSF), the radius of gyration (Rg), and solvent accessible surface area were analyzed. Further, the hydrogen bonds formed during simulation between the xylopic acid or rasagiline at the binding site of MAO-B were analyzed. Through the essential dynamics, two principal components (PC1 and PC2) were determined and used as reaction coordinates in identifying the metastable conformations of each complex through Gibb’s free energy surface (FES) analysis. The most unique conformations occupying the lowest energy basins were identified from Gibb’s FES. Cluster analysis was performed using the TTClust program [49, 50] to identify the most prominent conformations clustered in 10 clusters. The free energy of binding was analyzed from the end-state free energy calculation performed on the trajectories isolated at each 100 ps from the reasonably stable simulation period of 75 ns to 100 ns using the gmx_MMPBSA version 1.52 tool [51].

### 2.4. ADMET studies

ADMET is a technique utilized to examine the pharmacokinetic characteristics of a potential drug candidate. In this study, the pharmacokinetic property of the drug candidate was investigated using the admeSAR 2.0 online server [52]. The parameters examined include blood brain barrier permeability, solubility, human intestinal absorption, carcinogenicity and hepatotoxicity. Also, the drug likeness property of the drug candid was examined by considering the Lipinski’s rule of 5 (molecular weight ≤ 500, Log P ≤ 5, HBD (hydrogen bond donors) ≤ 5 and HBA (hydrogen bond acceptor) ≤ 10) [53].

## 3. Results and discussion

### 3.1. Molecular docking analysis

Molecular docking was employed to evaluate the MAO-B inhibitory property of Kaurane diterpenes from *X*. *aethiopica*. Rasagiline was used as the standard drug and its binding energy (-7.3 kcal/mol) was set as the cut off point to select the drug candidate **(Table 1).**

**Table 1:** Interaction analysis of xylopic acid in MAO-B binding pocket.

Ligands	Binding Energy (kcal/mol)	Hydrogen Bond Interaction		Hydrophobic Interaction	Pi-interaction
		Amino acid residue	Distance (Å)		
**Xylopic acid**	-9.3	Ser39	1.9132 2.9046	Tyr60, Leu171, Ile198, Phe343, Tyr398, Tyr435	Tyr60, Tyr343, Tyr398, Tyr435
		Tyr60			
**Rasagiline**	-7.3	-	-	Val294, Lys296, Phe343, Trp388, Tyr398	Val294, Lys296, Phe343, Trp388, Tyr398

A considerably high binding energy of -9.3 kcal/mol was obtained for xylopic acid, compared to rasagiline and that of the co-crystallized ligand that gave -8.4 kcal/mol. The oxygen atom on the kaurene diterpene moiety established two hydrogen bonding interactions with Ser39 at 1.9132 Å and Tyr60 at 2.9046 Å, compared to rasagiline that formed no hydrogen bonding (**Fig 1A**). Xylopic acid further strengthened its stability with the formation of hydrophobic interactions with Tyr60, Leu171, Ile198, Phe343, Tyr398, Tyr435, while rasagiline also established hydrophobic interactions with Val294, Lys296, Phe343, Trp388 and Tyr398 (**Fig 1B**). Pi-interactions were also established between the xylopic acid and Tyr60, Tyr343, Tyr398, Tyr435, while rasagiline also had pi-interactions with Val294, Lys296, Phe343, Trp388 and Tyr398.

**Fig 1:** Docked poses and interaction diagrams. A) xylopic acid MAO-B complex and B) rasagiline MAO-B complex.

Overall, xylopic acid and rasagiline formed common hydrophobic interactions with Phe343 and Tyr398, while common pi-interactions were observed with Tyr343 and Tyr398. Hydrophobic interaction contributes to the binding energy elicited in the binding pocket of the enzyme by xylopic acid and rasagiline, while the pi-interactions established helped to stabilize the phytochemical and standard drug at the receptor’s binding pocket. [54, 55] suggested that the addition of different substituents like carbonyl, hydroxyl and esters to the diterpene moieties and other phytochemicals could enhance their biological activities against diseases like diabetes, PD, malaria and allergies. This scenario is observed with xylopic acid such that the presence of the carboxylic acid group enhances the binding energy value obtained in the docking studies.

### 3.2. Molecular dynamics simulations

The RMSD in backbone atoms of MAO-B in apo form and complex with the standard drug rasagiline and xylopic acid showed lower deviations until around 20 ns (**Fig 2A**). There was a steep rise in RMSD thereafter, which remained almost stable until the end of the simulation period. The steep increase in the RMSD was due to the flip of an N-terminal helix in all the systems. The RMSD in backbone atoms of MAO-B remained relatively stable in the complex of xylopic acid after around 60 ns compared to the apo structure and the rasagiline complex. The RMSD in rasagiline and xylopic acid atoms remained almost constant, averaging around 0.06 and 0.07 nm, respectively (**Fig 2B**). Rasagiline has fewer atoms than xylopic acid. However, the lower and stable RMSD in the atoms of xylopic acid suggests it remained stable in the binding site.

**Fig 2:** MD analyses. A) RMSD in backbone atoms, B) RMSD in ligand atoms, C) RMSF in side chain atoms of residue, D) Radius of gyration, and E) Solvent accessible surface area analysis.

The RMSF analysis showed that compared to apo MAO-B, the rasagiline and xylopic acid complexes had more significant fluctuations in the residues range 50–60, 150–160, and 280–340 (**Fig 2C**). Particularly, MAO-B in the complex with rasagiline showed slightly higher fluctuations than the xylopic acid complex. Most of the residues in the above-mentioned ranges belong to the binding site, as the docking studies revealed. The more significant fluctuations in these residues signify the binding site adaptability to these ligands.

The radius of gyration analysis also showed initially more significant deviations until around 20 ns, which corroborates the lower RMSD in the backbone atoms of MAO-B in all the systems under study. In the case of MAO-B xylopic acid complex, after around 20 ns simulation period, the Rg lowers slightly until around 60 ns and remains stable and lowest compared to apo and complex with rasagiline (**Fig 2D**). The Rg in MAO-B rasagiline complex was lowered after around 20 ns; however, it deviated considerably until the end of the simulation. The Rg in apo MAO-B was also lowered after around 20 ns and remained stable with an average of 2.35 nm.

The SASA analysis showed that the xylopic acid complex had the lower SASA with an average of around 225 nm^2^ and remained almost stable and constant after around 70 ns (**Fig 2E**). On the other hand, the SASA for the rasagiline complex deviated considerably and stabilized after around 60 ns with an average of around 228 nm^2^. The apo MAO-B showed a larger SASA compared to the other two complexes, and interestingly after around 60 ns, the SASA was found to rise with an average of around 230 nm^2^. The larger the SASA, the more hydrophobic residues in deeper buried pockets are exposed to the solvent, resulting in the protein’s defolding or less stability [56]. Xylopic acid complex with lower SASA implies better stability of the corresponding complex.

The results of hydrogen bond analysis showed that xylopic acid formed more consistent hydrogen bonds (**Fig 3**). The results corroborate the docking results where the docked xylopic acid formed hydrogen bonds with Ser58 and Tyr60. With more nonbonded interactions, such as hydrogen bonds, and hydrophobic interactions, a ligand forms better in the binding affinity and ligand efficacy [57]. Xylopic acid formed more hydrogen bonds, reaching a maximum of 4 hydrogen bonds until around 25 ns, and thereafter, one hydrogen bond was formed consistently throughout the rest of the simulation. Unlike docking results, the equilibrated trajectory showed a single hydrogen bond with Ser59. However, this hydrogen bond is broken during simulation, and the trajectory at 25 ns showed four hydrogen bonds with Ile199, Gln206, Phe343, and Tyr326. Out of these, the bonds with Ile199 and Gln206 remained stable until 50 ns. The trajectories at 75 ns and 100 ns showed a hydrogen bond with Gly342 and Met341, respectively. In the case of standard rasagiline, a single consistent hydrogen bond was formed throughout the simulation, reaching a maximum of two in a few trajectories. However, no hydrogen bond is formed from 55 ns to around 95 ns in several trajectories. The equilibrated trajectory showed a hydrogen bond with Tyr398. The trajectory at 25 ns showed two hydrogen bonds with Leu171 and Cys172 residues. These hydrogen bonds broke at 50 ns, and the hydrogen bond with Tyr398 was again formed. The trajectory at 75 ns showed a new hydrogen bond with Tyr435 and trajectory at 100 ns reestablished the hydrogen bond with Leu171.

**Fig 3:** Hydrogen bond analysis.

The residues involved in hydrogen bond formation in each trajectory are difficult to identify, given the large size of the data. In this situation, the contact analysis where the contact frequency between the ligand and the residues within the distance of 0.35 nm, the most probable distance for a stable hydrogen bond, is valuable. The standard rasagiline showed more than 50% contact frequency with Gln206, Tyr398, Tyr435, and Gly434 and around 30% with Phe343 (**Fig 4A**). The residues Tyr398 and Tyr435, having higher contact frequency, have also been identified in hydrogen bond analysis. In the case of xylopic acid, Gln206, Phe343, Leu171, and Tyr326 had better than 50% contact frequency and Ile199 had better than 30% contact frequency (**Fig 4B**). Most of these residues, except Leu171, had also been identified in hydrogen bond analysis. The contact frequency analysis and hydrogen bond analysis results suggested that the residues Gln206 and Phe343 are important in rasagiline and xylopic acid.

**Fig 4:** Contact frequency analysis. A) MAO-B rasagiline complex and B) MAO-B xylopic acid complex. (Contact frequency determined for ligands at the distance of 0.35 nm).

After diagonalizing the covariance matrix for the C-α atoms in principal component analysis, the eigenvectors and eigenvalues or two principal components PC1 and PC2 were obtained [58]. These principal components were used as reaction coordinates in Gibb’s free energy analysis [59]. The results showed that the apo MAO-B metastable conformations exited in two low-energy basins (**Fig 5A**). The lowest energy basin occupied the region between -1.5 to -1 on PC1 and -1.5 to -0.8 on PC2, while another energy basin with slightly higher energy of 2 to 4 kJ/mol occupied the region -2.2 to -1.8 on PC1 and 1.2 to 2.0 on PC2. The representative metastable conformations from these energy basins differ in the N-terminal helix. In the rasagiline complex, metastable conformations existed in three low-energy basins (**Fig 5B**). If the values of PC1 and PC2 are high positive represents highly correlating conformations, while high negative values represent anti-correlating conformations. Out of the three energy basins, two energy basins existed in the correlating region. The energy basin occupying regions 1 to 2 on PC1 and 0.5 to 1.0 on PC2 had the lowest energy metastable conformations. However, the representative metastable conformation from this energy basin showed no key interactions between rasagiline and surrounding residues. The representative conformation from the other energy basin with slightly higher energy in the range 2.5 to 5.0 kJ/mol occupying the region 0 to 1 on PC1 and -2.5 to -1.5 on PC2 showed a hydrogen bond between rasagiline and Tyr398. The hydrogen bond analysis and contact frequency analysis also identified this residue as a key residue influencing the binding affinity of rasagiline. In the case of xylopic acid, two low-energy basins were found in the highly correlating region (**Fig 5C**). The representative metastable conformation from the smaller lowest energy basin occupying the region between 0.8 to 1.2 on PC1 and -1.7 to -1.2 on PC2 showed the hydrogen bonds between xylopic acid and residues Ile199, Gln206, and Met341. The hydrogen bond analysis and the contact frequency analysis also highlighted the importance of Ile199 and Gln206 residues in influencing the binding affinity. In addition to these residues, Gibb’s free energy analysis suggested that the residue Met341 could also result in the metastable lowest energy conformation. The other low-energy basin conformations showed no key interactions between xylopic acid and surrounding residues.

**Fig 5:** Gibb’s free energy analyses. A) Apo MAO-B, B) MAO-B rasagiline complex, and C) MAO-B xylopic acid complex. (The metastable conformations are shown for lowest energy basins for apo MAO-B where conformation in green belongs to energy basin I and conformation in red belongs to energy basin II. The respective conformations for MAO-B rasagiline complex and MAO-B xylopic acid complex are shown in respective figure panels).

The trajectories isolated at each 100 ps were clustered in 10 clusters to confirm the existence of stable conformations of respective complexes. In the case of rasagiline, the trajectories from 50 ns onward during the simulation period existed in four clusters, 7 to 10 (**Fig 6A**). The average structure from cluster 7 showed a hydrogen bond between rasagiline and residues Leu171 and Cys172. The average structures from the other three clusters had no key hydrogen bond interactions, where cluster 8 represented the most significant cluster. On the other hand, the xylopic acid complex showed three clusters, 8 to 10, existing after around 60 ns simulation period (**Fig 6B**). The average conformations of clusters 8 and 10 showed a hydrogen bond between xylopic acid and residue Ile199, while cluster 9 showed a hydrogen bond with residue Gln206. This further confirms these residues’ importance in better binding affinity of xylopic acid.

**Fig 6:** Cluster analysis. A) MAO-B rasagiline complex and B) MAO-B xylopic acid complex. (The average structures from select clusters are shown at the bottom of each figure panel).

The RMSD, RMSF, Rg and SASA analyses suggested the stability of xylopic acid MAO-B complex compared to rasagiline MAO-B complex and apo MAO-B. The hydrogen bond analysis pointed out that xylopic acid has a better propensity of forming hydrogen bonds at the binding site, while the contact frequency analysis further supported the hydrogen bond analysis. Gibb’s free energy analysis and cluster analysis also suggested that a larger number of xyloipc acid MAO-B complex conformations existed in the lowest energy states, and these conformations had the key hydrogen bond interactions.

The results of MM-GBSA calculations performed on the trajectories isolated at each 100 ps from the simulation period 75 ns to 100 ns are given in **Table 2.**

**Table 2:** MM-GBSA calculations.

Energy component (kcal/mol)	Xylopic acid	Rasagiline
ΔVDWAALS	-40.83 ± 2.14*	-27.52 ± 1.94
ΔEEL	-1.28 ± 0.39	-15.72 ± 2.49
ΔEGB	8.56 ± 0.42	19.26 ± 2.19
ΔESURF	-5.12 ± 0.13	-3.98 ± 0.17
ΔGGAS	-42.10 ± 2.08	-43.24 ± 2.55
ΔGSOLV	3.45 ± 0.38	15.28 ± 2.23
ΔTOTAL	-38.66 ± 2.10	-27.96 ± 1.87
-TΔS (Entropic contribution)	3.22 ± 0.05	2.55 ± 1.81
ΔG_Binding_	-35.43 ± 2.10	-26.15 ± 1.87

* Standard deviation

ΔVDWAALS: van der Waals energy; ΔEEL: Electrostatic energies; ΔEGB: Polar solvation energy; ΔESURF: Nonpolar solvation free energy; ΔGGAS = ΔVDWAALS+ΔEEL; ΔGSOLV = ΔEGB + ΔESURF; ΔTOTAL = ΔGSOLV +ΔGGAS; ΔG_binding_ = ΔTOTAL—TΔS

It is evident that xylopic acid has better free energy of binding (-35.43 ± 2.10 kcal/mol) than the rasagiline (-26.15 ± 1.87 kcal/mol). This is in part due to more favorable van der Waal’s interaction energy and considerably higher electrostatic interaction energy for the xylopic acid. The polar solvation free energy was slightly higher for rasagiline compared to xylopic acid.

### 3.3. ADMET studies

The identification of phytochemicals as MAO-B inhibitors depend on their ADMET and drug likeness properties. The ADMET property helps to predict the adsorption, toxicity, and metabolic potentials of hit molecules identified from computational, in vitro and in vivo studies [60]. In this study, the solubility, human intestinal absorption, blood-brain barrier, carcinogenicity and hetapotoxicity properties of xylopic acid were examined.

The solubility of and human intestinal absorption of xylopic acid gives useful information on its ease of dissolution and metabolism in subjects with PD. The blood-brain barrier permeability property of the drug candidate indicates its ability to cross the blood-brain barrier layer which is important for central nervous system based drugs. Xylopic acid showed good human intestinal absorption and solubility properties. Solubility values ranging between -6.5 to 0.5 are acceptable for a drug candidate [61, 62]. Also, Xylopic acid exhibit BBB permeability, indicating that it exibit potential to penetrate the brain tissue of PD subjects.

In terms of toxicity, the ADMET profiling indicated that xylopic acid was neither carcinogenic nor hepatotoxic when taken by PD subjects. AMES toxicity test is used to predict the mutagenic potential of phytochemicals [60, 63]. The result of the AMES test showed that xylopic acid exhibit no toxicity. The hERG I and II (human Ether-a-go-go-Related gene) helps to control the ion channels implicated in the heart’s cardiac electric action potential [32]. In this study, xylopioc acid showed no hERG I and II inhibition. Furthermore, the oral rat acute toxicity (LD_50_), oral rat chronic toxicity, skin sensation and minnow toxicity showed that the compounds is safe and within the acceptable limit. Additionally, the ligand obey the drug likeness principle based on Lipinski’s rule of 5, whereby their molecular weight < 500, hydrogen bond acceptor ≤ 10, hydrogen bond acceptor ≤ 5, Log P < 5 (Lipinski).

## 4. Conclusions

In this present study, molecular docking studies were used to identify xylopic acid as potential MAO-B inhibitor. Molecular dynamics simulation was employed to understand the binding mode, interaction and estimate the binding free energy of the phytochemical in the binding pocket of MAO-B. ADMET studies were used to evaluate the pharmacokinetic properties of xylopic acid. The phytochemical elicited good binding affinity with the MAO-B compared to the standard drug. The potential drug candidate formed hydrogen bonding, hydrophobic and pi-interactions which enhanced its stability at the enzyme’s binding pocket. Xylopic acid established good binding energy in the molecular dynamics simulations compared to the standard rasagiline. The ADMET and drug likeness studies suggested xylopic acid to be a potential drug candidate against the MAO-B enzyme. In the ADMET studies, xylopic acid showed good blood-brain barrier permeability property and solubility in the gastrointestinal tract which is good for an antidepressant agent. The study posited xylopic acid as a potential drug candidate in the treatment of PD. Comprehensive in vitro studies are recommended for future studies.

## Supporting information

S1 Fig Chemical structures of kaurane diterpenes. (DOCX)
